The article "Resource Allocation Strategy of the Educational Resource Base for MEC Multiserver Heuristic Joint Task" was published in 2022. Journal: Comput Intell Neurosci.

# Resource Allocation Strategy of the Educational Resource Base for MEC Multiserver Heuristic Joint Task

**DOI:** 10.1155/2022/4818767

**Published:** 2022-05-14

**Authors:** Ning Luo

**Affiliations:** School of Intelligence and Information Engineering, Guangxi Economic and Trade Vocational Institute, Wuzhou, Guangxi 520021, China

## Abstract

This paper analyzes the application of MEC multiserver heuristic joint task in resource allocation of the educational resource database. After constructing the scenario of educational resource database, a mathematical model is constructed from the dimensions of local execution strategy, unloading execution, and given educational resource allocation, in order to optimize the optimal allocation of educational resources through MEC. The results show that the DOOA scheme has good performance in terms of calculation cost and timeout rate. Compared with other benchmark schemes, the DQN-based unloading scheme has better performance, can effectively balance the load, and is better than the random unloading scheme and the SNR-based unloading scheme in terms of delay and calculation cost. The results show that the total hits of all category 1 users' content requests account for the proportion of the total content requests. The images have a small downward trend at the 15000 and 30000 time slots and then continue to rise. This shows that the proposed scheme can automatically adjust the caching strategy to adapt to the changes of content popularity, which proves that the agent can correctly perceive the changing trend of content popularity when the popularity of network content is unknown and improve the caching strategy accordingly to improve the cache hit rate. Therefore, the allocation of educational resources based on the MEC multiserver heuristic joint task is more reasonable and can achieve the optimal solution.

## 1. Introduction

With the rapid development of computers and information technology, mankind has entered the information age. Beginning with the national events, the leaders of the China Information Ministry presented the idea of China's information reform to the context of the country's information network, information technology, technology and business, knowledge of technology, and the rules of technology, rights, and patterns. The structure is shown in Figure 1. For the information construction of an industry, information networks are the foundation, information resources are the core, the use of information and the use of information technology is the goal, and information talents, information technology industry, and information policies, regulations, and standards are its guarantee [1, 2].

With the rapid growth of educational resources and applications, the requirements for cloud infrastructure and wireless access networks are becoming higher and higher. In order to provide communications, IT, and cloud computing services directly from the learning edge, the concept of mobile edge computing was adopted. Different from the traditional education resource database computing system, the MEC server is the host of the network operator and can be used directly at the mobile terminal or in the wireless area accessed by the corresponding computer, which allows MEC to make applications closer to end-users, reducing end-to-end latency and alleviating the backhaul network load [3–5].

With the emergence of MEC, resource-limited mobile devices can offload computing tasks to MEC servers, thus enabling them to support the services and applications of various educational resource libraries, such as network education, Internet of Things education system construction, and educational image processing. Task offloading generates additional overhead in latency and energy consumption due to communication between the device and the MEC server in the uplink wireless channel. Furthermore, in the system with a large number of educational users, the limited computing resources on the MEC server severely affect the task execution delays. Therefore, performing resource allocation becomes a key issue for achieving efficient computational offloading.

## 2. Literature Review

Due to the differences in economic and social development, the degree of educational informatization varies greatly, and there are also major differences in the development of education and services. Teachers in American schools are highly informed, and the curriculum is usually developed by the teachers themselves. Only a few teaching auxiliary software (such as Blackboard, Angle, life text, WebCT, U-Learn, and Illuminate) have been developed by the Ministry of Education in combination with universities or research institutions. User resource service modes mainly include the following: (1) The Internet-based free download form of service is only provided by a few sources, and the type and amount of resources are minimal, often some courseware, magazines, and other resources. For example, the famous MIT (Massachusetts Institute of Technology) advocates the OCW (open courseware) movement, which translates the courseware of many courses into different language versions and publishes them online for people around the world to learn for free. (2) Online ordering of resources in the form of e-commerce and transmission by mail or express delivery are mainly limited to educational software and educational courseware. This form accounts for a certain proportion in European and American countries with a sound social security system. In the United States, many educational resource banks accept credit card payments. As long as the funds of the user account are guaranteed, they can quickly obtain specific educational resources. Educational resources include both K12 resources for basic education and various professional resources, such as health care, aerospace, history, and culture. (3) The vast majority of service users use the web portal as a simple presentation format, with a friendly and easy-to-find interface, which can provide timely services, such as research documents and frequently asked questions. Many portals can be configured for different credentials to provide different functions. For example, the Eric resource library supported by the U.S. Department of Education includes not only complete database content services for group users (such as some schools and scientific research institutions) but also customized and personalized resource services for individuals according to their needs. The portal related to Eric asks Eric, which contains rich Eric resources and can provide timely resource services for teachers, librarians, consultants, managers, and parents.

At present, the development of China's educational resource pool is still at an embryonic node, and there are many disadvantages in the distribution of the educational resource pool. The coupling of edge computing systems (MEC) and educational resource databases will greatly improve the rational allocation of educational resources. Based on the measurement of edge technology, the problem of allocating resources can be divided into three categories: single-user edge technology, multiuser edge technology, and heterogeneous server edge computing system. The following introduces the research status of these three types of resource allocation problems:

1. Single user edge computing system: considering the utilization efficiency of educational resources, the single user multiserver edge computing system is generally not considered. Because its utilization rate of educational resources is very low, the single user edge computing system generally refers to the system composed of an edge device and an edge server. In order to obtain the conditions for computing unloading, Nouri et al. modeled the computing time and communication time at the same time and obtained the completion time of the task in the two cases of local computing and unloading to the server computing [6]. Previous studies have shown that if only the delay is considered, unloading can be considered when the delay of local calculation of the task is higher than that of unloading it to the server for execution. In order to obtain the relationship between the edge computing system parameters and the offload task parameters, Shi et al. introduced two parameters CCR (computing to communication ratio) and RLR (remote to local ratio) to analyze the conditions of computing offload and obtained the inequality between CCR and RLR. Assuming that the communication system is in the nonblocking case, the queuing delay and forwarding delay are removed. Finally, the inequalities of edge computing system parameters and computing task parameters are obtained. This inequality can be used as a reference formula for unloading decision-making. Only computing tasks that meet this inequality can be unloaded to the edge server for execution [7]. Huang et al. studied the problem of minimizing the energy consumption of mobile devices under the constraint of given completion time, as shown in Figure 2. Computing tasks generated by edge devices are either executed locally or unloaded to the server for execution [8]. The author assumes that the tasks are indivisible and can only be unloaded completely. When the computing task is executed at the server, only the energy consumption of wireless communication needs to be considered [9]. In this paper, the author proposes a framework to minimize the energy consumption of edge devices in random wireless channels. When the computing task is executed in the edge device, the CPU energy consumption is minimized by dynamically adjusting the clock frequency. When the computing task is executed at the server, the wireless communication energy consumption is minimized by adjusting the wireless transmission power of the edge device. By solving these two scheduling problems, the optimal unloading decision is obtained [10].
2. Multiuser edge computing system: multiuser edge computing system generally refers to a system composed of multiple users and an edge server. Educational resources and wireless communication resources are centrally allocated by edge servers. In order to solve the problem of centralized educational resource allocation, the author first abstracts the joint wireless and computing resource optimization problem into a convex optimization problem by establishing a wireless communication model and computing model, and then obtains the solution of the convex optimization problem by the Lagrange multiplier method. In addition, the author also concludes that there is a one-to-one mapping relationship between the transmission energy allocated to each channel and the number of CPU cycles allocated to relevant users and proposes a license control strategy. Its core idea is to allow the tasks to be transmitted to the edge processing and the disallowed tasks to be processed locally, which can not only ensure that the edge server is not overloaded but also ensure the stability of the task queue of the edge device [11, 12]. The definition of an educational resource allocation problem is that the edge equipment performs the educational resource allocation process, while the definition of a centralized educational resource allocation problem is that the server performs the process. The author first models the allocation problem of educational resources and wireless resources then formalizes it into a multiuser unloading game problem and proves that the unloading game problem has Nash equilibrium. Based on this, the author announces the distribution of electronic components and obtains the maximum limit on the assembly time and the total cost of the system. The experimental results show that, compared with other algorithms, the total cost of this algorithm; that is, the weight of the delay and the power consumption are reduced by at least 51%.
3. Heterogeneous server edge computing system: heterogeneous server edge computing system generally refers to a system composed of multiple servers and multiple edge servers. Some studies have added cloud servers to this system to form an end edge cloud three-tier architecture. Consider a three-tier system architecture composed of edge devices, edge cloud, and remote cloud, in which the edge cloud is composed of multiple edge servers. Due to the limited computing and storage capacity of the edge cloud, the competition of educational resources among multiple users should be considered. The author uses queuing theory to establish a multiuser resource competition model to obtain user interaction information and the impact of computing offload on user perception performance. Then, according to the model, the author formalizes the multiuser resource competition problem into a generalized Nash equilibrium problem, also known as noncooperative game problem. Based on the in-depth analysis of the equilibrium problem, a distributed equilibrium algorithm suitable for the problem structure is proposed. The experimental results show that the response time delay is reduced by more than 20% compared with other methods [13].

Based on this research, an overall solution is developed in a multiMEC server-assisted network to optimize the distribution of learning groups, hence maximizing user offloading results. The electrical offloading of each user is the first model based on the weight of the finished time and the energy consumption of the equipment; then a combination of offloading operations and the allocation of training resources is designed as a nonlinear integrated system, transforming the complex problems of the first into a cohesive system. Finally, the goal of collaborative work to improve user experience and user uplink transmission is achieved by using the low-stress heuristic algorithm planned in the form of this text.

## 3. Method

### 3.1. Construction of Educational Resource Database Scene

Considering the two-layer heterogeneous UDNS scenario enabled by the MEC, as shown in Figure 3, the system model is composed of one macro base station (MBS) and K small base station (SBS). MBS connects with SBS through the wired link and controls the association scheme and educational resource allocation between user equipment (UE) and SBS by collecting information such as educational resource storage, channel quality status, and user task attributes of SBS. The set of SBS is represented as *k* = {1, 2,…, *K*}. Each SBS is equipped with an ES, and the UE associated with the same SBS-ES pair shares the resources on the base station side, including wireless resources and educational resources. The UE set is expressed as *n* = {1, 2,…, *n*}. Each UE has a computing-intensive task that needs to be completed within the specified time limit. The computing task can be executed locally on the UE or completely unloaded to any SBS-ES pair for processing. Each terminal can only select one SBS for association and unload the computing task to the corresponding ES [14, 15].

Define the binary variables *φ*_*nk*_={0,1}, ∀*n* ∈ *N*, and *k* ∈ *K* as the associated variables. If UE *n* selects to be associated with SBS *k*, then *φ*_*nk*_=1; otherwise *φ*_*nk*_=0.

Therefore, ∑_*k*∈*K*_*φ*_*nk*_=1 indicates that the UE selects any SBS for task unloading, while ∑_*k*∈*K*_*φ*_*nk*_=0 indicates local processing of computing tasks. The task model of UE *n* can be described as TASK_n_ = {*d*_*n*_, *ω*_*n*_, *T*_*n*_^max^, *α*_*n*_, *β*_*n*_}. Among them, *d*_*n*_ is the large input file of the operating system and *ω*_*n*_ is the computer equipment required to complete the computer operation, and the number of CPU cycles used as much as possible case. *T*_*n*_^max^ is the maximum tolerable delay of the task. Because different UEs have different task requirements, UEs with small battery capacities want lower energy consumption, while UEs sensitive to task delay want lower processing delay. Therefore, the calculation cost is defined as the weighted sum of delay and energy consumption, and *α*_*n*_ and *β*_*n*_ are weighting factors indicating the attention of different UEs to delay and energy consumption. Specifically, UE can be divided into four categories according to UE itself and its task attributes.

If the computing task of the UE is time delay sensitive but the battery capacity of the UE is large enough, then *α*_*n*_ = 1 and *β*_*n*_ = 0.5 indicate that the UE has higher requirements for time delay than the equipment energy consumption [16, 17]. The reason why it is set to 0.5 instead of 0 is that we still want to pay some attention to the equipment energy consumption rather than completely ignore the energy consumption of this kind of UE. However, compared with other UE that pay more attention to the equipment energy consumption, it is necessary to reduce the weight of this kind of UE in the item of energy consumption. On the contrary, if the UE battery capacity is limited and wants to reduce equipment energy consumption and have a high tolerance for task delay, make *α*_*n*_ = 1, and *β*_*n*_ = 1. The reason is the same as above. Similarly, if UE has high requirements for delay and energy consumption, *α*_*n*_ = 0.5, *β*_*n*_ = 0.5, UE has loose requirements for both [18].

The number of resources on the SBS side can be described as Res_*k*_ = {*B*_*k*_, *F*_*k*_, *E*_*k*_}, where *B*_*k*_ is the available bandwidth of SBS *k* and *F*_*k*_ is the maximum computing power of ES *k* (unit: CPU cycles/second). Since SBS uses green energy as the main energy source, *E*_*k*_ is the green energy storage of SBS *k*. This paper considers the quasi-static scenario and assumes that the green energy reserve of SBS is a fixed random value in a scheduling cycle, and the energy consumption of SBS should not exceed its energy reserve. For each UE, the maximum transmit power and local CPU cycle frequency are expressed as *P*_*n*_ and F_*n*_^l^, respectively.

### 3.2. Calculation Model

Local execution strategy: in order to save power, it is assumed that UE can dynamically adjust CPU frequency and voltage by using DVFS technology according to the different requirements of tasks on computing power. *f*_*n*_ refers to the local computing capacity of UE *n*, in CPU cycles/s. Since there is no transmission delay for local execution, the local execution delay is the same as the calculation time in the following formula:

(1) $$\begin{array}{c} t_{n}^{l}=\frac{\omega_{n}}{f_{n}}. \end{array}$$

The energy consumption of one CPU cycle can be modeled as *k*(*f*_*n*_)^2^, where *k* is the effective conversion capacitance, and its value depends on the chip structure. Therefore, the total energy consumption of UE is shown in the following formula:

(2) $$\begin{array}{c} e_{n}^{l}=kf_{n}^{2}\omega_{n}. \end{array}$$

Unloading execution: if the UE decides to unload the task to any SBS-ES, the unloading execution delay includes uplink transmission delay, calculation delay, and downlink transmission delay. Since the results of computing tasks are usually very small, the downlink transmission delay can be ignored. UE associated with the same SBS allocates orthogonal spectrum, so there is no intra cell interference between UE which is associated with the same SBS. [19–21]. The uplink transmission rate is shown in the following formula:

(3) $$\begin{array}{c} r_{nk}=B_{nk}\log_{2}\left(1+\frac{h_{n,k}P_{n}}{N_{0}B_{n,k}}\right), \end{array}$$

where *B*_*nk*_ represents the channel bandwidth allocated by SBS *k* to UE *n*, *P*_*n*_ represents the transmission power of UE *n*, *h*_*nk*_ is the channel gain between SBS *k* and UE *n*, and *N*_0_ is the power spectral density. Therefore, the uplink transmission time of transmission task data *d*_*n*_ can be calculated by using the following formula:

(4) $$\begin{array}{c} t_{n}^{l}=\frac{d_{n}}{r_{nk}}. \end{array}$$

Given the educational resource allocation *f*_*n,k*_; that is, the number of calculated educational resources allocated by ES *k* to its associated UE *n*, the calculation time of task TASK_*n*_ is:

(5) $$\begin{array}{c} t_{n}^{c}=\frac{\omega_{n}}{f_{n,k}}. \end{array}$$

The unloading execution delay can be obtained from the above two items:

(6) $$\begin{array}{c} t_{n}^{0}=t_{n}^{u}+t_{n}^{c}. \end{array}$$

Similarly, the transmission energy consumption and calculation energy consumption of the UE task unloading can also be calculated. The uplink transmission energy consumption of UE *n* is shown in the following formula :

(7) $$\begin{array}{c} e_{n}^{0}=P_{n}t_{n}^{u}. \end{array}$$

The calculated energy consumption of ES *k* processing task TASK_*n*_ is shown in the following formula:

(8) $$\begin{array}{c} e_{n,k}=\omega_{n}\delta , \end{array}$$

where *δ* is the energy consumption of ES per CPU cycle. This paper assumes that the total energy consumption of SBS is mainly composed of two parts: static energy consumption Ε_*k*_^*0*^ and calculated energy consumption. Where Ε_*k*_^*0*^ represents the energy consumed by SBS *k* to remain active without traffic load. The calculated energy consumption is the total energy consumed by executing the calculation task of the associated UE. Note that the total energy consumption of SBS cannot exceed its energy reserve, this is also shown in the following formula:

(9) $$\begin{array}{c} {Ε}_{k}^{0}+\sum_{n=1}^{N}\varphi_{n,k}e_{n,k}\leq E_{k}. \end{array}$$

To sum up, the total execution delay of task TASK_*n*_ can be expressed as following formula:

(10) $$\begin{array}{c} t_{n}=\sum_{k=1}^{K}\varphi_{n,k}t_{n}^{0}+\left(1-\sum_{k=1}^{K}\varphi_{n,k}t_{n}^{0}\right)t_{n}^{l}. \end{array}$$

## 4. Result Discussion

Figures 4 and 5 show the average value of the calculation and the operating time of the system with the change of UE. It can be seen that the average price calculation and time discount of the four strategies increase with the increase of UEs, and the DOOA strategy is better than the other three ideas with the two measures above.

The user association distribution of the three unloading schemes is shown in Figures 6–8. The circular area in the figure represents the cell, taking the location of the cell center MBS as the origin, and the abscissa and ordinate, respectively, represent the horizontal distance and vertical distance relative to the origin, in meters [22, 23]. In the figure, the Pentagon represents SBS, scattered points represent UE, different colors are used to distinguish, which SBS-UE is associated with, and the number in the legend in the upper right corner represents the number of UE associated with different SBS. It can be seen from the figure that under the random unloading scheme, UE is completely randomly distributed in the whole coverage area. In the SNR-based unloading scheme, UE is closely distributed around SBS, which leads to an uneven distribution of UE. The number of UE associated with SBS in hot spot areas is more, while the number of other SBS is relatively lower. In the unloading scheme based on DQN, the quality status of Beixiao and the distribution of educational resources are comprehensively considered, and the distribution of users is more decentralized and uniform than that based on SNR. The number of associations under different SBS is more average, and it is also superior to the random unloading scheme. The UE associated with the same SBS are evenly distributed around the SBS, unlike the random scheme scattered in the whole spatial range, and the spatial span between UEs is large.

Figures 9 and 10 show the total delay and calculation cost of each SBS of the three schemes, respectively. As shown in the figure, the unloading scheme based on the DQN can effectively realize load balancing. Compared with other unloading schemes, the delay and calculation cost of each SBS have a smaller variation range and are more average. Due to its random characteristics, the random unloading scheme makes the number of associations of each SBS relatively uniform and can effectively balance the load. However, due to the fact that a random scheme completely does not consider the information such as user task attributes and base station resource distribution, the random scheme has poor performance compared with the scheme based on the DQN. It can be seen from the figure that the DQN scheme has better performance in terms of delay and calculation cost, both of which are significantly lower than the random scheme, as shown in SBS in Figure 9.

The simulation results show that the unloading scheme based on DQN makes full use of the task attributes of UE and the distribution of SBS educational resources to divert UE, so as to achieve a better unloading strategy and potentially achieve load balancing. The SNR scheme based on the proximity principle cannot effectively balance the load to obtain good performance, and the random scheme has the worst performance.

In addition, all users want to get a good service experience, and there are two heterogeneous services competing for limited storage and educational resources in the network. Improper resource allocation will lead to unfairness among heterogeneous users. For example, when the edge node SBS caches a large amount of user content, the hit probability of content requests will increase significantly, which will improve the service experience of class 1 users, but this will occupy the storage space of the computing offload service, and the number of computing offload users acceptable to SBS will decrease significantly, and vice versa. In order to ensure the fairness between heterogeneous service users as much as possible, the scheme HOMC proposed in this section considers three points to coordinate the use of storage resources by two types of users. Firstly, due to the lag effect of the cache strategy, the cache decision is always made before the unloading decision. The proposed cache strategy based on MADDPG predicts the storage space required for unloading the service in the next time slot based on the total size of all current class 0 user task data in each time slot, makes the cache decision, and updates the cache. For the proposed heuristic unloading strategy, SBS gives priority to providing unloading services for users with a small amount of computing task data in each time slot to accommodate more user access. In addition, a penalty item is also introduced into the reward function to avoid over updating the cache. When the cached content changes more, the penalty is greater, which also avoids the excessive occupation of storage resources by the edge cache.

In order to measure the impact of educational resource allocation on the fairness of heterogeneous users, Figure 11 shows the fairness factors in the training process. The change curve of *R* shows that *Z* gradually rises and tends to be stable, which means that the proposed model can try to ensure fairness between the two types of users after training.

Because the proposed caching scheme does not know the content popularity in advance but learns the content popularity change trend according to the user's content request, so as to make the caching decision. In order to verify the adaptability of the proposed caching scheme based on MADDPG to the change of content popularity, Zipf distribution is used to generate user content requests, and the content in the network is renumbered every 15000 time slots to change the content popularity. The ordinate in Figure 12 is the cumulative cache hit rate, which is defined as the proportion of the total hits of all class 1 user content requests to the total content requests up to the current time. It can be seen that the image has a small downward trend at the 15000 and 30000 time slots and then continues to rise, which shows that the proposed scheme can automatically adjust the caching strategy to adapt to the changes of content popularity. It is proved that when the popularity of network content is unknown, the agent can correctly perceive the changing trend of content popularity and improve the caching strategy to improve the cache hit rate.

## 5. Conclusion

The integrated optimization problem of offload input and distribution of class resources in MEC-enabled dual-layer heterogeneous UDNS is studied, and the basic process is designed to solve optimization problems. Firstly, the system model in the current scenario is described, and the corresponding computing models are described, according to whether the user task is executed locally or unloaded. Then, a hybrid optimization problem of joint unloading strategy, transmission power, computing resources, and bandwidth allocation is formed with the goal of minimizing the system computing cost under the constraints of limited resources and QoS guarantee. In order to solve the complex optimization problem, a DOOA scheme is proposed, which decouples the unloading strategy from the resource allocation sub problem and solves it in two stages. In the first stage, an improved algorithm based on DQN is used to determine the unloading scheme, and in the second stage, alternating optimization and the Lagrange multiplier method with KKT constraints are used to solve the problem of educational resource allocation. The simulation results show that the DOOA scheme has good performance in terms of calculation cost and timeout rate. Compared with other benchmark schemes, the DQN-based unloading scheme has better performance, can effectively balance the load, and is better than the random unloading scheme and the SNR-based unloading scheme in terms of delay and calculation cost.

## Figures and Tables

**Figure 1:** Information architecture.

**Figure 2:** Cloud-assisted mobile application platform.

**Figure 3:** System model.

**Figure 4:** Average calculation cost of the system.

**Figure 5:** System average timeout rate.

**Figure 6:** Distribution of users in DRL mode.

**Figure 7:** User distribution in SNR mode.

**Figure 8:** User distribution in random mode.

**Figure 9:** Total delay of each SBS in three schemes.

**Figure 10:** Calculation cost of each SBS of three schemes.

**Figure 11:** Impact of education resource allocation on the fairness of two types of users.

**Figure 12:** Impact of content popularity change on cache hit rate.

## Data Availability

The labeled datasets used to support the findings of this study are available from the corresponding author upon request.
